# Monitoring and Model Analysis of Vocal Performance Teaching Environment Using Cluster Analysis from the Perspective of Core Literacy

This article has been retracted.

**DOI:** 10.1155/2022/1477309

**Published:** 2022-10-06

**Authors:** Tao Long

**Affiliations:** School of Arts, South China University of Technology, Guangzhou 510006, China

## Abstract

To cultivate students' artistic quality, enhance their vocal music quality, and prepare them to make great contributions to the innovation and development of my country's vocal music art is the main goal of opening vocal music performance major in colleges and universities. With the advancement of technology and the demands of talent development, the vocal music teaching methodology for the vocal music performance major in colleges and universities must be continuously enhanced. Otherwise, there will be an issue of disconnect between teaching style and talent development, which will harm both the development of high-quality vocal music talents and the innovation and growth of vocal music performance majors in colleges and universities. The vocal music performance major at colleges and universities should actively support the reform and innovation of the vocal music teaching mode in order to extend students' knowledge, develop their all-around ability, and provide a strong foundation for vocal music performance, to develop students' all-encompassing musical abilities. This research suggests a design strategy for the monitoring and model optimization of the teaching environment for vocal performance majors from the standpoint of core literacy. To increase the efficiency and objectivity of course instruction, cluster analysis aids students in categorising and searching for vocal music performance main repertoire as well as using collaborative filtering recommendations to locate their own vocal music performance. The simulation test analysis is completed lastly. The method has a certain accuracy, which is 7.59% higher than the conventional algorithm, according to the simulation findings. In addition to significantly increasing student interest in studying vocal music performance courses, we further reform and innovation of the teaching method for these courses at colleges and universities can also strengthen students' understanding of various repertoire styles and significantly enhance their musical literacy.

## 1. Introduction

With the reform of national policies, the curriculum reform of basic education has mainly turned to a new stage aimed at improving the core quality of students [1]. Unlike the previous teaching paradigm based on the presentation of teaching content, curriculum and teaching pay more and more attention to the cultivation of students' comprehensive ability and quality [2]. The three basic components of the students' development core quality are cultural foundation, independent growth, and social participation. The material of this core quality is highly rich. Through the creation and realisation of various quality indicators, it seeks to enable students to acquire the necessary character and key ability to meet the needs of future society development and solve comprehensive problems under various situations. The proposal of the core quality of the vocal performance discipline is a major adjustment in the concept of the vocal performance curriculum reform. Therefore, we can regard the cultivation of students' cultural understanding literacy as the new goal of vocal performance teaching [3]. The core accomplishment of pursuing cultural understanding is not to regard vocal music performance as an art or a technology but to regard vocal music performance as “an understanding of specific society, culture and history, reflecting the characteristics, abilities, and levels of cultural creation of a country and a nation.” This concept is not only consistent with the overall trend of studying vocal music performance as a cultural phenomenon in the anthropology of vocal music performance, but also closely related to the understanding of culture, integrity, and relevance in art from the perspective of ecological civilization [4]. Through the study and practice of the vocal performance course, students cultivate and develop their perception of sound, explore its cultural connotation, understand the vocal performance works and vocal performance phenomena from a cultural perspective, and finally form the cultural understanding ability of vocal performance [5]. The cultivation of this ability will also become the main direction of the reform and efforts of the vocal performance course at present and in the future [6].

The creative subject of vocal music performance is the performer himself. The teaching purpose of this course is to train the performance skills of the singer, give full play to his personality, and create his own vocal music artistic image with his unique voice color and performance method. With the efficient interconnection of the Internet, more and more data will be transmitted and used by users. In the face of broad application scenarios, more and more recommendation arithmetics are regarded as very effective and important information technology solutions [7–9]. The basic idea of collaborative filtering recommendation is to find the highest rated items from the user neighborhood set of similar users and then recommend the items to the target users after ranking and calculating to a certain extent. The recommendation arithmetic based on collaborative filtering has the advantage that it can analyze the content of music, movies and other machines that cannot automatically analyze their content. At the same time, it can find and recommend new information in time, obtain potential but unknown content of users, recommend more personalized content, and effectively use user feedback information. The approach of similarity score in collaborative filtering is used in this research to lower the execution cost of the arithmetic because of the benefits of collaborative filtering arithmetic. It has been demonstrated via practise that this combination not only speeds up calculations but also enhances the effectiveness of teaching vocal performance as a specialty.

The vocal performance training course adopts the method of combining theory with practice. By learning the basic theoretical knowledge of vocal music performance, analyzing and processing vocal music works, training performance skills and skills, and cultivating the interest and desire of performance, students can strengthen their stage control, improve their performance skills, and further improve their vocal singing ability with the help of performance. So that students of professional courses can fully achieve the combination of singing and performance, better adapt to, and be competent for singing performance in various artistic practices, extracurricular program arrangement activities and vocal music teaching and research work that may be faced in the future [10]. The establishment of vocal performance training courses is in line with the current prosperity and development of cultural undertakings and the needs of the art talent market. The exploration and research on this course also have strong practical value [11]. This paper establishes a feature reconstruction model for the teaching optimization design of vocal music performance specialty, searches the tracks suitable for the vocal music performance by clustering arithmetic, studies the personalized music by collaborative filtering arithmetic, and extracts the fuzzy features of the teaching optimization design of vocal music performance specialty. Its innovation lies in the following:

1. In this paper, the method of similarity score in collaborative filtering is used to reduce the execution cost of the arithmetic
2. This paper constructs the key feature quantity of the teaching optimization design of vocal music performance specialty and uses cluster analysis to realize the teaching optimization design and identification of vocal music performance specialty

## 2. Related Work

“Core” mainly reflects the following characteristics in the presentation of music literacy: basic, irreplaceable, and general [12]. Vocal performance belongs to stage art practice. Any practical activity must have strong theoretical support and be guided by scientific and systematic theoretical knowledge and effective laws and methods. The specific links included in vocal performance training are various, and the knowledge and theories related to lines, singing, music, body, and performance also need to be studied [13].

Zheng et al. put forward targeted implementation suggestions on the development of students' vocal core quality from the nature, objectives, contents, and basic concepts of junior and senior high school vocal music courses [14]. DFSABC combines the educational value brought by the vocal music course with the vocal music practice. After investigation and analysis, it puts forward the strategy of implementing the core quality of students' development in the basic education stage [15]. Joer et al. studied the connection between the core accomplishment and the singing teaching part of the junior high school vocal music course and considered that the “three-dimensional goals” of emotion, attitude, values, process and method, knowledge, and skills are the basis of the core accomplishment [16]. Bertollo and others introduced the origin of core literacy and the development of various countries, regions, and organizations in detail. From an international perspective, this paper makes a comparative analysis of the core literacy indicator systems of the United States, France, Britain, and Japan. Based on the profound traditional culture, we also explored the indicators suitable for the development of students' core literacy and conducted detailed research and analysis on how to implement them [17]. Kiehel and Falkenbach combined theory with practice. Through abundant teaching cases, this paper introduces the specific ways and methods of cultivating students' core literacy in classroom teaching, emphasizes that teaching reform must start from changing teaching concepts, and expounds in detail the transformation of knowledge teaching to literacy teaching [18]. Mohammed et al. elaborated the concept of vocal music curriculum based on the understanding curriculum paradigm in detail. They believed that the philosophical basis of the understanding paradigm of vocal music curriculum was hermeneutics, phenomenology, and the philosophy of vocal anthropology and that the proposed curriculum paradigm was a breakthrough and challenge to vocal music as a universal “scientific system” [19]. Hasnain et al. proposed that the scientific understanding theory, humanistic understanding theory, and practical understanding theory of vocal music are all of great importance to vocal music education. Each has its own advantages and limitations, and the three complement each other [20]. Lee et al. put forward that understanding classroom practice requires that curriculum teaching is a dialogue and communication activity based on the curriculum text. As far as the teaching class is concerned, the cultural understanding paradigm of vocal music teaching advocates a teaching strategy towards intersubjective understanding and communication [21].

To sum up, the research content related to the vocal music course under the core competence has become more and more diversified, and the understanding of related issues has become more and more in-depth. At the same time, from the perspective of the research in the field of vocal music, the direct literature is relatively rare, which also provides a large academic space for this paper to carry out relevant research. This paper puts forward an optimization design scheme of the teaching mode of the vocal performance professional course in the perspective of core accomplishment and studies the personalized music of the vocal performance professional course in combination with clustering analysis and collaborative filtering arithmetic, so as to optimize the course teaching from the aspects of formulating personalized performance tracks and make the professional course teaching more scientific.

## 3. Methodology

### 3.1. Using Clustering Arithmetic to Screen Vocal Music Performance Tracks

The selection of vocal music repertoire is a thorough representation of the vocal abilities and levels of vocal music learners. Each vocalist possesses a certain voice type and set of performance skills. The right song selections will help vocal music teachers maximise their students' potential and steadily advance their vocal music abilities. Music has the qualities of rich variation, huge number, quick listening duration, coherence, and order; thus, the accuracy of music classification cannot be solved by using classic single arithmetic. Data mining technology has emerged as one of the greatest options to address these issues as a result of the production of large amounts of data and the rapid development of artificial intelligence and information technology. Cluster analysis technology, which is at the foundation of data mining, is continually improving and iterating thanks to deeper study, more innovative ideas, better optimization techniques, and a wider range of research topics.

Researchers are still looking at three crucial technologies: feature representation, feature extraction, and matching arithmetic, in order to improve the retrieval effectiveness and precision in content-based music retrieval. As a result, the cluster class containing the cluster center with the highest similarity is chosen after the music pieces to be matched are first matched with each cluster center. The music that has to be matched is then successfully matched with every song in the cluster. Before retrieval, the music database's audio features are grouped, and the center of each cluster is identified and saved in the feature database. Studies show that employing this strategy can drastically reduce retrieval times while simultaneously ensuring a high level of retrieval accuracy. The MIDI format songs from the database are used as the object for the hierarchical clustering of the music collection together with the foundations of *K*-means hierarchical arithmetic. The implementation strategy for hierarchical clustering employed in this work is shown in Figure 1.

The specific implementation steps of the arithmetic are as follows:

1. Firstly, the MIDI file is extracted from pitch and length, and the feature database is established
2. In the feature database, the feature of a song is randomly selected as the first cluster center, and the similarity between other candidate song sets and the cluster center is compared by using the one-sided continuous matching method. The candidate song sets with the same similarity and the highest similarity are grouped into a cluster together with the cluster center, and the cluster center *k*_1_ is marked
3. The music piece with the minimum similarity value in the above comparison is taken as the next cluster center. If there are several minimum values, one music piece is randomly selected as the cluster center *k*_2_ of the second cluster. And it calculates the similarity between the remaining music pieces in the feature library and the cluster center, classifies the candidate song sets with the same similarity and the highest degree together with the cluster center into a cluster, and marks the cluster center *k*_2_
4. The loop steps (2) and (3) cluster the remaining songs to form different clusters and mark the cluster centers of each cluster until each song is included in each cluster
5. The music pieces with correct melody are accurately matched with the songs in the music library, and the matching results are output. The accuracy and practicability of clustering are verified by the accuracy and search efficiency

The appeal method is based on the hierarchical clustering method, which discards the restrictions of *K*-means arithmetic on the number of clusters and the center points of clusters, and makes the clustering results more objective. The flow chart of hierarchical clustering arithmetic is shown in Figure 2.

In clustering arithmetic, the similarity measurement between sample data is a very important link, and distance is often used as a classification statistic in clustering analysis. According to the data characteristics of this paper, a similarity measurement method based on one-sided continuous matching arithmetic is adopted. When clustering data objects, data objects are first regarded as points in space, so the distance between data objects can be regarded as the distance between points. Assuming that the objects *x*_*i*_, *y*_*j*_ are all data objects with *p* dimensional attributes, the distance formula between the description objects *x*_*i*_ and *y*_*j*_ should meet the following conditions:

1. Nonnegativity: that is, the distance between any two objects *i*, *j* is always *d*_*ij*_ ≥ 0, and only when the *p* attribute variables of the two objects are equal, *d*_*ij*_ ≥ 0 holds
2. Symmetry: that is, for all any two objects *i* and *j*, there is always *d*_*ij*_ = *d*_*ji*_
3. Trigonometric inequality: that is, for all three arbitrary objects *i*, *j* and *k*, there is always *d*_*ij*_ ≤ *d*_*ik*_ + *d*_*kj*_

The distance measurement formula satisfying the above three conditions can make the distance between two objects within the range of [0, ∞). The smaller the distance, the closer the two objects are, and the more similar their properties are. The commonly used distance definitions in cluster analysis include Euclidean distance, Manhattan distance, Chebyshev distance, and Mingshi distance. Specific definitions are as follows:

1. Euclidean distance:

(1) $$\begin{array}{c} d_{ij}={\left(\overset{p}{\underset{k=1}{\sum }}{\left(x_{ik}-x_{jk}\right)}^{2}\right)}^{1/2}. \end{array}$$

(2) Manhattan distance:

(2) $$\begin{array}{c} d_{ij}=\overset{p}{\underset{k=1}{\sum }}\left|x_{ik}\right.-\left.x_{jk}\right|. \end{array}$$

(3) Chebyshev distance:

(3) $$\begin{array}{c} d_{ij}=\underset{1\leq k\leq p}{\max}\left|x_{ik}\right.-\left.x_{jk}\right|. \end{array}$$

(4) Mingshi distance:

(4) $$\begin{array}{c} d_{ij}={\left(\overset{p}{\underset{k=1}{\sum }}{\left(x_{ik}-x_{jk}\right)}^{q}\right)}^{1/q}. \end{array}$$

The Mingshi distance is the general formula of some distance functions. At *q* = 2, the Mingshi distance is Euclidean distance; at *q* = 1, the Mings distance becomes Manhattan distance; at *q* = ∞, the Mings distance is the Chebyshev distance.

### 3.2. Search for Vocal Performance Music Based on Collaborative Filtering Arithmetic

The key abilities in the core literacy include information processing ability, reflective thinking ability, communication and coordination ability, and innovation and creation ability. Under the background of the network era, there are many network resources such as music network platform, music website, and music network course. In their interaction, students have basically realized the ability to use new media such as computers and mobile phones to process information such as words, audio, images, and videos. Some even use modern information to perform music and other activities.

There is a tonne of knowledge available because to the Internet and information technology's quick development. Our personal needs have been greatly enriched by this information, but it has also resulted in the issue of information overload. The recommendation system was created in order to better address the users' unique needs and address the information overload issue. The collaborative filtering arithmetic is one of the most often used arithmetic in the music recommendation system. The target user's habits and interests are taken into account while evaluating items using this arithmetic, and the user is then given recommendations for relevant products. The relevant data that users filled out on questionnaires or in the user's browsing or purchasing history could also count as historical information. The collaborative filtering-based recommendation algorithm has great personalization and can automatically identify users' potential areas of interest, which steadily enhances the system's effectiveness in terms of recommendations. Tables 1 and 2 demonstrate the benefits and drawbacks of the centralised recommendation arithmetic.

The performance of the recommendation system is influenced by the quality of its construction model, which forms the basis of the link between the computing resources of the system. One of the most established and extensively used personalized recommendation systems is collaborative filtering recommendation arithmetic.

Assuming that the user set is represented by *U*, *I* represents the set of items, and the recommendation degree of the item *i* to the user *u* can be expressed by the function *S*, and the recommendation arithmetic can be expressed in the form of

(5) $$\begin{array}{c} \forall u\in U,i=\arg\max S_{ieI}\left(u,i\right). \end{array}$$

The performance of recommended arithmetics is usually measured according to some authoritative evaluation standards. This section briefly summarizes the commonly used evaluation standards of recommended arithmetics.

The method used to calculate recommendation prediction scores is now the most popular. In order to infer and anticipate the user's scores on other items, a comparable model is typically created based on the user's historical data. When assessing how well the arithmetic performs, the average absolute error and root mean square error are the most crucial calculating techniques. In general, the closer the result is near the true value and the higher the quality of the arithmetic's recommendation, the smaller the two values are.

(6) $$\begin{array}{c} \text{MAE}=\frac{\sum_{\left(u,i\right)\in T}\left|r_{ui}-f_{ui}\right|}{\left|T\right|},\\ \text{RMSE}=\frac{\sqrt{\sum_{\left(u,i\right)\in T}{\left(r_{ui}-f_{ui}\right)}^{2}}}{\left|T\right|}, \end{array}$$

where *T* represents the test set, *r*_*ui*_ represents the actual score of the user on the item, and *f*_*ui*_ represents the predicted score of the user on the item.

In addition, accuracy and recall are typically taken into account simultaneously in the comparison study of suggested findings. The percentage of correctly suggested items among all items is represented by the accuracy rate. Recall rate is the percentage of recommended things in the total number of favourable items provided by the target user; the higher the recall rate, the more accurate the recommendation. The recommendation's accuracy increases as the value increases. The accuracy and recall equation is as follows:

(7) $$\begin{array}{c} \text{Precision}=\frac{\sum_{u}\left|R_{u}\cap T_{u}\right|}{\sum_{u}\left|R_{u}\right|},\\ \text{Recall}=\frac{\sum_{u}\left|R_{u}\cap T_{u}\right|}{\sum_{u}\left|T_{u}\right|}, \end{array}$$

where *u* is the user, *R*_*u*_ is the actual recommendation result, and *T*_*u*_ is the test recommendation result.

Since the arithmetic cannot take into account the results of both at the same time to a great extent, the weighted average value, i.e., *F*_1_ value, is usually taken for the results of both according to the actual situation:

(8) $$\begin{array}{c} F_{1}=\frac{2*\text{precision}*\text{recall}}{\text{precision}+\text{recall}}. \end{array}$$

In addition, the recommended evaluation indicators include coverage, diversity, novelty, surprise, robustness, and user satisfaction.

## 4. Result Analysis and Discussion

The layered teaching method is the most commonly used teaching mode in the vocal performance class of colleges and universities at present. It refers to the application of the latest scientific and technological means, combined with the objective factors such as students' learning ability, vocal performance foundation, and progress space, to carry out group layered guidance. If we want to find a direction suitable for the development of music students, we must first make education and teaching face all students, give play to students' individual characteristics, give full play to their strengths and avoid their weaknesses, teach students according to their aptitude, and improve and enrich teaching concepts, teaching models, teaching systems, and teaching methods suitable for social development and students' knowledge reserves.

The hit rate and retrieval impact of the subsequent retrieval validate the accuracy of the clustering in light of the properties of the music in the music library. Both this method and the traditional approximate symbol matching arithmetic are employed for the retrieval under the aforementioned circumstances. The effectiveness and superiority of the retrieval method in this research are confirmed through the hit rate of the retrieval. The clustering of two notes, or the approximate symbol matching arithmetic, is the linear superposition of their pitch and length differences, and it employs the proper transfer cost to indicate the melody change brought on by the addition or subtraction of notes.  Figure 3 displays the approximate symbol matching and clustering arithmetic's retrieval hit rates.

The first hit rate was 65%, the first four hit rates were 75%, and the first 15 hit rates were 94% after clustering. The approximation symbol matching arithmetic has a first 15 bit hit rate of 85%, first four bit hit rate of 62%, and first bit hit rate of 60%. The application arithmetic after clustering offers clear advantages in the average retrieval hit rate, as can be observed in Figure 4.

For various note numbers, the system's retrieval speed varies. The retrieval time for 20 notes in a music library containing 4000 songs is typically around 15 seconds, while the retrieval time for 7 notes is around 10 seconds, according to the experimental findings of the authors of the Lam arithmetic. According to Figure 4, using the lam arithmetic after clustering takes just a sixth as long as using the lam arithmetic alone for a music collection of the same size. After using the music clustering arithmetic based on one-sided continuous matching, the running time of music retrieval is only approximately 2–5 seconds if the size of the music library is around 10,000 pieces.

In order to verify the difference in accuracy, recall and *F*_1_ value between collaborative filtering recommendation based on tag fusion time factor, collaborative filtering recommendation based on user interest and collaborative filtering recommendation combined with traditional collaborative filtering recommendation, the accuracy and feasibility of the new arithmetic are verified. According to the classic “two eight principle,” 80% of the data set is selected as the training set, and the remaining 20% is selected as the test set. After many experiments, it is found that the length of the recommendation set also has an impact on the experimental results. Therefore, the length of the recommendation set *n* is set to 0-30. The reason for this is that the length of the recommendation set is too short to be representative, and the calculation time required for the recommendation set is too long, and the user may be upset. Therefore, it is very important to set an appropriate length of the recommendation set. For the tag collaborative filtering recommendation arithmetic with time factor, a control test is set, and the traditional user-based collaborative filtering recommendation and the item based collaborative filtering recommendation are taken as the control group. The experimental results are shown in Figures 5–7.

Figure 5 shows the comparison between collaborative filtering recommendation based on users and articles and the recommendation accuracy of tags fused with time factors. It can be seen intuitively that the overall recommendation accuracy decreases with the increase of recommendation set length, but the recommendation effect of tags fused with time factors is better than those of the other two traditional collaborative filtering recommendation arithmetics.

In Figure 6, the collaborative filtering suggestion based on users, the collaborative filtering recommendation based on articles, and the recommendation recall rate of the tags fused with the time factor are compared. The recommendation effect of the tags fused with the time factor is better than those of the other two conventional collaborative filtering recommendation arithmetic, despite the intuitive observation that the total recommendation recall rate improves with the length of the recommendation collection.

Figure 7 shows the results of combining the accuracy rate and recall rate of F1 values of the three arithmetics. It can be seen that they all show a trend of rising first and then falling.

In this chapter, the three arithmetics mentioned above are tested, and then, the results are analyzed. First, the experimental data set is selected, and lastly, in the FM data set, 80% of the experimental set is used as training and 20% is used as test set. In terms of the accuracy, recall, and *F*_1_ value, the recommendation based on the fusion time factor, the recommendation based on the user's interest, and the traditional collaborative filtering recommendation arithmetic based on users and articles are compared in the form of a broken line graph. It can be seen clearly and intuitively that the new arithmetic has improved the performance of various indicators; that is, the recommendation performance has certain advantages.

## 5. Conclusion

The teaching method for the vocal music performance specialty is presented in this paper as an optimised design scheme from the standpoint of core literacy. In order to increase the efficiency and objectivity of the course instruction, it aids students in categorising and searching the tracks of the vocal music performance specialty through clustering analysis, and it uses collaborative filtering recommendation to find their own vocal music performance. The simulation test analysis is completed lastly. According to the simulation results, the proposed arithmetic is 7.59% more accurate than the conventional arithmetic in terms of precision. This result fully demonstrates that the problems in collaborative filtering arithmetic are properly solved by combining the concepts of hierarchical clustering arithmetic and collaborative filtering arithmetic. One-sided continuous matching arithmetic is used to calculate the similarity value between musical pieces. As a result, the clustering outcomes are tolerable and offer the best data support for subsequent matching retrieval. Through experimental analysis and verification, it can be seen that the general concept of research and improvement is more workable, the math works successfully and effectively, and the results are to some extent improved compared to the original math. From the vantage point of teaching methodology and curriculum execution, it is the advancement of education and teaching concept to pay attention to the training of vocal performance professionals. It is important to continuously test and refine the analysis and research on the vocal music performance training programme in real-world settings. The course's standardised design and ideal environment will contribute to better preparing singers with strong vocal abilities and those working in related cultural and artistic fields. In this paper, the improvement of collaborative filtering arithmetic is limited. In fact, there are still problems of cold start and scalability. The cold start problem can be solved by using hybrid recommendation.

## Figures and Tables

**Figure 1:** Implementation block diagram of hierarchical clustering arithmetic.

**Figure 2:** Flow chart of hierarchical clustering arithmetic.

**Figure 3:** Retrieval hit rate of Lam arithmetic and approximate symbol matching arithmetic after clustering.

**Figure 4:** Average time consumption of Lam arithmetic and Lam arithmetic after clustering.

**Figure 5:** Precision value of each arithmetic.

**Figure 6:** Recall value of each arithmetic.

**Figure 7:** *F*_1_ value of each arithmetic.

**Table 1:** Advantages of various recommended arithmetics.

Content based recommendation	Collaborative filtering recommendation	Recommendation based on association rules	Recommendation based on deep learning
(1) The recommendation result is relatively direct	(1) With the accumulation of data, the accuracy of recommendation becomes higher	(1) Can handle unstructured data	(1) Strong ability to learn from samples
(2) Easy to understand and do not require unique domain knowledge	(2) Recommended personalization	(2) It effectively solves the problem of data sparsity	(2) The models are rich
(3) There is no data sparsity problem	(3) Increased automation	(3) Effectively improve the cold start problem	(3) Rich recommendations
	(4) Able to handle complex unstructured data	(4) Handle the association between data	(4) It can fuse all kinds of scenario data

**Table 2:** Disadvantages of various recommended arithmetics.

Content based recommendation	Collaborative filtering recommendation	Recommendation based on association rules	Recommendation based on deep learning
(1) Cold start of new users	(1) Cold start of new projects	(1) Rely on a large amount of data	(1) There are problems such as cold start and sparse data
(2) Complex attributes are difficult to handle	(2) Data sparsity	(2) Application limitations	(2) The optimization of the model and the degree of its effect are to be discussed
(3) Domain knowledge required	(3) Cold start of new users	(3) The more rules there are, the more irrelevant rules there are	(3) Under certain circumstances, new resources of interest cannot be found for users

## Data Availability

The data used to support the findings of this study are available from the corresponding author upon request.
